# Breast Cancer Diagnosis by Convolutional Neural Network and Advanced Thermal Exchange Optimization Algorithm

**DOI:** 10.1155/2021/5595180

**Published:** 2021-11-08

**Authors:** Xiuzhen Cai, Xia Li, Navid Razmjooy, Noradin Ghadimi

**Affiliations:** ^1^Community Health Service Center, Taibei Street, Jiangan District, Wuhan, 430010 Hubei Province, China; ^2^Wuhan Vocational College of Software and Engineering, Wuhan, 430205 Hubei, China; ^3^Department of Engineering, Tafresh University, Tafresh, Iran; ^4^Young Researchers and Elite Club, Islamic Azad University, Ardabil Branch, Ardabil, Iran

## Abstract

A common gynecological disease in the world is breast cancer that early diagnosis of this disease can be very effective in its treatment. The use of image processing methods and pattern recognition techniques in automatic breast detection from mammographic images decreases human errors and increments the rapidity of diagnosis. In this paper, mammographic images are analyzed using image processing techniques and a pipeline structure for the diagnosis of the cancerous masses. In the first stage, the quality of mammogram images and the contrast of abnormal areas in the image are improved by using image contrast improvement and a noise decline. A method based on color space is then used for image segmentation that is followed by mathematical morphology. Then, for feature image extraction, a combined gray-level cooccurrence matrix (GLCM) and discrete wavelet transform (DWT) method is used. At last, a new optimized version of convolutional neural network (CNN) and a new improved metaheuristic, called Advanced Thermal Exchange Optimizer, are used for the classification of the features. A comparison of the simulations of the proposed technique with three different techniques from the literature applied on the MIAS mammogram database is performed to show its superiority. Results show that the accuracy of diagnosing cancer cases for the proposed method and applied on the MIAS database is 93.79%, and sensitivity and specificity are obtained 96.89% and 67.7%, respectively.

## 1. Introduction

Breast cancer is common cancer and is the first cause of cancer mortality in women. Breast cancer is a malign tumor that develops from cells in the same organ. The disease usually begins in the lobules, or breast ducts, and can then penetrate the ducts and walls of the glands and attack the surrounding adipose tissue or even other parts of the body. There may be other lumps in the breast that are not cancerous, but in any case, the final diagnosis is up to the physicians. Science has proven that despite the existence of a way to prevent cancer and the lack of definitive treatment for this disease, early diagnosis of this disease helps physicians to at least prevent the progression of this disease. The number of cancer patients in the world is increasing. Based on the World Health Organization (WHO), breast cancer has a great effect on about 2.1 million women annually. Based on this statistic, in 2018, 627,000 women have died of breast cancer which contains about 15% of all deaths among women cancer [1].  Figure 1 shows the statistical information of the cancer diagnosis and the cancer deaths in 2019 [2].

The best solution to decline breast cancer mortality is to diagnose it in the primary stage and treat it. Early diagnosis needs a precise and dependable diagnostic method. Among the various methods of diagnosing breast cancer, mammography is a very common and very popular method. Systematic screening of the female population with mammograms and early diagnosis of early stage breast cancer can also increase the patients' survival chances and reduce the negative side effects of necessary treatments. These results are possible if the quality of services is provided in the best possible way.

On the other hand, the diagnosis of breast cancer based on mammography film has several problems. In some cases, there is a possibility that the film is damaged or the image is not suitable for diagnosis. Meanwhile, the film wears out over time, and the possibility of revision decreases. On the other hand, the only tool a doctor can use to diagnose a lesion is a visual video. The physician's visual observations to diagnose the lesion leads to two errors. The first is that a radiograph is shown twice to a physician or radiologist. If he does not know that both images are the same, his diagnosis may be different. Another error is showing an image to two physicians or two radiologists, each of whom has a different diagnosis. Although mammography is usually the best way to diagnose breast cancer, some classes of cancers are not diagnosed in this way. In this condition, providing the computer-aided systems can detect malignant lesions efficiently [1]. Based on the literature, the effectiveness of a computer diagnostic system is more precise than that of a physician. Recently, various kinds of research works were performed in the area of the automatic early detection of breast cancers [3]. In other words, the higher efficiency of the computer-aided systems assists the physicians to diagnose cancer with lower complexity and higher speed. For instance, Liu et al. [4] proposed a proper image segmentation methodology for optimal breast cancer diagnosis regarding the interval uncertainties. For considering the indeterminacy, interval assessment was utilized. The method is guaranteed to providing suitable results in any changes in the imaging system. The main idea was to provide an interval-based Laplacian of Gaussian filter to simulate the intensity uncertainties. Final results have been performed to MIAS database, and a comparison of the results with some classic techniques was carried out to illustrate the method efficiency.

Toğaçar et al. [5] introduced a breast cancer diagnosis system by CNN. The method was improved by a technique called BreastNet. The image data was established by the expansion technique before implementing it into the model. Then, a precise classification method was accomplished based on the hypercolumn technique. Then, a comparison of method results with some latest techniques was done to state the higher precision of the suggested system.

Carvalho et al. [6] used another method for breast cancer detection for utilizing in histopathological images. The authors presented a method for using phylogenetic diversity indexes to determine images to model creation and histopathological breast image classification into some classes. The method was then compared with several different latest techniques to demonstrate the technique's accuracy. The results showed significant robustness to the method to help experts at large medical centers.

It can be concluded from the previous studies that many works have been done for the automatic diagnosis of breast cancer. This paper proposes a new automated method for breast cancers diagnosed in mammogram images. Here, an optimized deep learning-based methodology based on a new improved metaheuristic, called Advanced Thermal Exchange Optimization algorithm, has been used for this purpose.

## 2. Image Preprocessing

The heterogeneity of light intensity in medical images has weakened the boundaries of medical images, especially the heterogeneity of light intensity in magnetic resonance images created by nonuniform magnetic fields by radiofrequency coils, which is why preprocessing is so important in medical research. Therefore, after obtaining the input information of the medical images, preprocessing operations should be performed, which are methods to eliminate noise and isolate and improve the differentiation of areas where there is a possibility of numerical information.

### 2.1. Image Contrast Improvement

Commonly, in images, several forms of contrast issues are existing, for instance, the inappropriate lighting and room conditions, the deficiency of enough applicant interface for imaging, and the inadequate quality of the measuring sensors and devices. These variables will disappear with some essential details, darkening or overexposure, and finally the image abnormalities. The presence of these variables increases their need for enhancement in numerous medical images. Lack of these parameters in most numbers of medical images increases their requirement for improvement. This improvement has been performed based on contrast enhancement.

Here, the contrast enhancement has been applied to the images to highlight the skin cancer areas with no changes on the other areas. A simple application to perform a piecewise linear contrast stretch operation on an image. The present study uses a 16-bit lookup table to improve the contrast of the images that are then stored on a disc. This is implemented based on the following formula:

(1) $$\begin{array}{c} y_{\text{hist}}=\frac{x_{\text{hist}}-{\mathrm{Min}}_{\text{hist}}}{{\mathrm{Max}}_{\text{hist}}-{\mathrm{Min}}_{\text{hist}}}, \end{array}$$

where Max_hist_ and Min_hist_ stand for the highest and the lowest levels for the gray magnitudes of the main image histogram, respectively, and *x*_hist_ and *y*_hist_ represent the input image before contrast enhancement and the output image after image contrast enhancement, respectively.

### 2.2. Noise Reduction

As aforementioned, due to different conditions in the medical imaging, there are some kinds of noises in them that should be removed before processing. This is done by using noise reduction. Noises can be white, random, or Gaussian (that contains a large part of medical images). Noise is usually in the high-frequency bands of the image; the important edges and details of the image are in the same bands. Therefore, noise removal along with preserving the edges and important image information is the main problem in the image noise removal process. Many noise removal techniques have been proposed in recent years. One of the proper methods for noise removal in medical images is to use the Wang-Mendel algorithm. This algorithm is a beneficial technique based on fuzzy theory [7]. Because of the simple conception of the fuzzy theory, the method of the Wang-Mendel algorithm is so easy to understand. Also, due to the higher speed of this method, it is too valuable for initial fuzzy model creation [8]. The method for the rule database is achieved by the following:

1. Perform fuzzy separation from the input variable space which can be obtained based on the knowledge or using normalization technique. Afterward, it classifies it into two parts including equal or unequal by performing a fuzzy separation of the input variable space. Afterward, the membership function has been selected and the components have been given as a fuzzy package. Afterward, membership has been chosen and a fuzzy set is given to every part
2. Creation candidate language rules which can be formed by choosing the most all-encompassing laws for the samples
3. Level of validity assignment to the laws that are achieved based on multiplying the membership function values of the components and the membership function value of the result of the law
4. Provide final database rules from the collection of candidate language which is done by classifying the candidate rules into various groups, where each of them contains candidate rules with similar assumptions. For obtaining the final rule base, the maximum degree of verification law is achieved in every set

## 3. Image Segmentation

### 3.1. Changing Color Space

However RGB has a good concept for the human, it is completely dependent on the three colors (red, green, and blue), as base colors of the RGB color space. This color space has also a high dependency on the ambient light intensity which limits its usages in a different application. To recover this issue, different color spaces have been introduced. In this study, the XYZ color space is utilized for the purpose after some trials and errors. The XYZ color space makes a link between the physiologically supposed colors in human color vision and distributions of wavelengths in the visible spectrum of the electromagnetic. In the XYZ color model, *Y* states the luminance, and *X* and *Z* indicate the color information. The formula for converting the RGB to XYZ is as follows:

(2) $$\begin{array}{c} \left[\begin{array}{c} X\\ Y\\ Z \end{array}\right]=\frac{1}{0.17697}\times \left[\begin{array}{ccc} 0.49 & 0.31 & 0.2\\ 0.17697 & 0.8124 & 0.01063\\ 0 & 0.01 & 0.99 \end{array}\right]\times \left[\begin{array}{c} R\\ G\\ B \end{array}\right]. \end{array}$$

The most significant benefit of the XYZ color model is that it is completely independent of the device.

### 3.2. Method of Segmentation

The red (*R*) color space provides the main dimension in RGB color space to give nearly the image intensity in medical images. As previously mentioned, both *X* and *Z* values provide similar color information for the XYZ color space. So, for segmentation, *X* dimension and red dimension are only normalized, i.e.,

(3) $$\begin{array}{c} \hat{R}=\frac{R}{\sqrt{R^{2}+G^{2}+B^{2}}},\\ \;\hat{X}=\frac{X}{\sqrt{X^{2}+Y^{2}+Z^{2}}}. \end{array}$$

These normalization values are carried out on every pixel in the input images. The Otsu threshold is used after this normalization to provide a low-cost segmentation in the sense of time complexity.

By intergroup variance optimization and lessening pixels' intragroup variance, the Otsu process is an efficient way that is established to automatically pick the optimal threshold. There is an issue with the global threshold when the resolution of the image background is insufficient. To remove the heterogeneity effect, it is possible to use a local threshold. To remove inhomogeneity and add a global threshold to the processed image, this problem is solved by image preprocessing.

Based on the Otsu method, the threshold value has been searched which minimizes the class-in-between variance as follows:

(4) $$\begin{array}{c} \sigma_{\omega }^{2}\left(t\right)=\omega_{1}\left(t\right)\sigma_{1}^{2}\left(t\right)+\omega_{2}\left(t\right)\sigma_{2}^{2}\left(t\right), \end{array}$$

where *ω*_*i*_ describes the probability for two different groups with a threshold magnitude of *t* and *σ*_*i*_^2^ represents the variance amount of the groups. In other words, Otsu indicates that variance minimization of a class is like maximization of the variance in class-within, i.e.,

(5) $$\begin{array}{c} \sigma_{b}^{2}\left(t\right)=\sigma^{2}-\sigma_{\omega }^{2}\left(t\right)=\omega_{1}\left(t\right)\omega_{2}\left(t\right){\left[\mu_{1}\left(t\right)-\mu_{2}\left(t\right)\right]}^{2}, \end{array}$$

where *μ*_*i*_ describes the mean value. The Otsu algorithm will be defined as the following pseudocode.

Subsequently, for better performance, postprocessing mathematical morphology, including filling, closing, and opening, was carried out on the images [9]. First, extra holes in the image are filled by applying the mathematical filling operator. The analytical model is as follows:

(6) $$\begin{array}{c} X_{k}=\left(X_{k-1}⊕B\right)\cap A^{c},\;k=1,2,3\cdots , \end{array}$$

where *A* and *B* describe the area that should be processed and the constructing element, respectively.

Afterward, the mathematical opening has been employed to the filled image to eliminate the ignitor information with no adjustments on other gray surfaces. The mathematical model of this operator is as follows:

(7) $$\begin{array}{c} A\circ B=\left(A⊖B\right)⊕B. \end{array}$$

Then, the mathematical closing is executed based on the following equation for linking the narrow parts:

(8) $$\begin{array}{c} A\cdot B=\left(A⊕B\right)⊖B. \end{array}$$

This study uses a 5 × 5 identity matrix as a structural element.  Figure 2 gives some examples of the breast segmentation of images depending on the approach suggested.

## 4. Feature Extraction

Feature extraction is the process of reducing the dimensional of the images by dividing and reducing an initial set of images to more controllable groups. So, the next processing of the images can be simpler by this process. Of these large datasets, the most important characteristic is that they have numerous parameters. To process them, these parameters need many calculating origins. Therefore, extraction of these features helps to select and combine variables into features to get the best feature from those big datasets, thereby effectively decreasing the data volume. In this study, two popular features including DWT and GLCM were employed for feature extraction that is described subsequently.

### 4.1. Discrete Wavelet Transform (DWT)

Wavelet transform is an efficient tool for various applications in image processing and is utilized in numerous fields such as image noise removal, pattern recognition, coding, image compression, and feature extraction. Wavelet transform is a method in the frequency domain. In this method, instead of using sine and cosine functions (such as Fourier transform), a function called wavelet is used. When implementing a wavelet transform, the wavelet function retains its shape but is displaced along with the signal and compressed and opened during the displacement, thus encapsulating the entire signal. Unlike short-time Fourier transform, this method can create different resolutions for low- and high-frequency ranges.

There are various solutions for implementing DWT, the most common of which is the implementation of Multiresolution Analysis (MRA). In this method, the implementation of discrete wavelet transform is done with the help of a series of consecutive operations that each step of this operation includes signal filtering and downsampling. At each stage of the discrete wavelet process, the signal content is decomposed into two orthogonal subspaces including a low-pass filter (LL) and a high-pass (HH) filter [10], which is then split into four classifications: LH, LL, HH, and HL.

To increase the frequency resolution, this decomposition is rendered consecutively, such that the approximation signal is passed through a pair of high- and low-pass filters and decomposed into two new information and approximate signals. Afterward, the read rapidity was reduced by 50 percent. To give more information, the HL subbands with further efficiency are applied. This process is mathematically formulated as follows:

(9) $$\begin{array}{c} P_{dwt}\left(s\right)=\left\{\begin{array}{c} d_{i,j}=\sum f\left(s\right)\times H*i\left(s-2\times i\times j\right),\\ d_{i,j}=\sum f\left(s\right)\times L*i\left(s-2\times i\times j\right), \end{array}\right. \end{array}$$

where *d*_*i*,*j*_ signifies the feature of the component in signal *f*(*s*), *L* and *H* describe the coefficients of low-pass and high-pass filters, respectively, and *i* and *j* stand for the wavelet and the translation factor scales, respectively.

### 4.2. Gray-Level Cooccurrence Matrix

To study the structure of different tissues, Haralick has proposed properties based on the GLCM, which is one of the most successful methods for studying the properties of different tissues [11]. In the gray surface cooccurrence matrix method, it is assumed that the texture image information is determined by a specific matrix. This method is relied on manipulating the gray surfaces of an image. In this method, in addition to examining the gray surface of the desired pixel, the gray surfaces of its neighboring pixels are also examined, and by creating a new matrix of gray surfaces of the pixel neighbors at different angles and distances, the image properties are identified and defined. The coevent matrix is a square matrix and its size is the amount to the gray surfaces' number.

The cooccurrence matrix of an image is defined using radius *d* and angle *θ*. Usually, *d* is selected in the range of 1 and 2. Since each pixel has 8 neighbors at *θ* equal to 0, 45, 90, 135, 180, 225, 270, and 315 degrees to define the cooccurrence matrix, so the angle selection may be up to 4 adjacent pixels at *θ* equal to 0, 45, 90, 135, and 180 degrees (horizontal, right diagonal, vertical, and left diameter). In addition to the radius and angle parameters used to define the cosmopolitan matrix, the gray number parameter can also be defined. In this study, to define the cooccurrence matrix, a radial distance of 1 with four zero angles and the number of 256 gray surfaces were used, for which a new matrix was extracted. Subsequently, the information about the utilized characteristics was explained. The first characteristic is *Contrast* that describes the intensity magnitude of the pixels and their neighborhood. The second feature is *Entropy* which defines the image selected interference. The third feature is *Energy* that describes the repetitive pixel pair quantity. The fourth feature is *Correlation* that defines the spatial feature reliance among the pixels. Finally, *Homogeneity* as the last feature as a local uniformity feature creates multiple/single intervals for accusing the nontextured/textured characteristics.  Table 1 indicates five gray-level cooccurrence matrix features extracted from the samples.

## 5. Convolutional Neural Networks

After feature extraction from the segmented images, they should be classified properly as the final step of diagnosis. In this study, convolutional neural network (CNN) was used for this purpose. CNNs are significant deep learning techniques where several layers are prepared strongly. This technique is very effective and is a usual technique in different applications of computer vision. An outline of convolutional neural network architecture is depicted in Figure 3.

Generally, a CNN is made of three major layers: the convolutional layer, the pooling layer, and the fully connected layer. Various layers do various tasks. Each convolution neural network includes two stages: feedforward and backward for preparation.

In the first step, the features enter the network, and this operation is the point multiplication between the input and the variables of each neuron, and finally, the application of convolution operations in every layer.

The output of the network is then computed. Here, to establish the variables related to network training, network output results are applied to compute the network error rate. To do this, a comparison of the network output to the correct solution (optimal solution) is carried out by an error function and the error rate is computed. In the later phase, by the computed error rate, the postrelease phase begins. The gradient of each variable is computed in this phase based on the chain rule, and all variables are altered by the influence they have on the error created in the network. Following parameters' updating, the feed-forward phase starts. Afterward, repeating a good number of these phases, the network preparing finishes. In this study, CNN is employed for local feature extraction in breast mammogram images. To offer optimum weighting among network connections, the backpropagation technique has been established. As the activation mechanism, a rectified linear unit (ReLU) is used.

With multiplying filter matrices by the images, feature maps are generated. To generate the feature map, the filter moves from left to right and up to down with a specific stride size to extract high-level features (like edges) until it finishes the full width. Here, the Max-pooling process uses the maximum value of the matrix in the feature maps to decrease the output neurons and the cross-entropy loss value based on backpropagation, which is formulated as follows:

(10) $$\begin{array}{c} L=\overset{\text{N}}{\underset{\text{j}=1}{\sum }}\overset{\text{M}}{\underset{\text{i}=1}{\sum }}-d_{j}^{\left(i\right)}\log\;z_{j}^{\left(i\right)},\\ d_{j}=\left(0,\cdots ,0,\underset{k}{\underset{⏟}{1,\cdots ,1}},0,\cdots ,0\right), \end{array}$$

where *d*_*j*_ signifies the proper output vector and *z*_*j*_ determines the achieved output vector for the *m*^th^ class. The softmax function is achieved as follows:

(11) $$\begin{array}{c} z_{j}^{\left(i\right)}=\frac{e^{f_{j}}}{\sum_{i=1}^{M}e^{f_{i}}}, \end{array}$$

where *M* describes the sample number.

To adjust function followed by keeping higher values, a weighting penalty (*ρ*) is added that is illustrated in the following equation:

(12) $$\begin{array}{c} L=\overset{\text{N}}{\underset{\text{j}=1}{\sum }}\overset{\text{M}}{\underset{\text{i}=1}{\sum }}-d_{j}^{\left(i\right)}\log\;z_{j}^{\left(i\right)}+\frac{1}{2}\rho \underset{K}{\sum }\underset{L}{\sum }W_{k,l}^{2}, \end{array}$$

where *W*_*k*_ defines the weight of connections and *L* and *K* define the overall number of layers and the layer *l* connections, respectively.

The CNN layouts were usually used based on trials and errors, which yielded inaccurate results. Numerous automated and optimized works have been implemented to address this problem [12]. The use of metaheuristic algorithms is one of the normal approaches. A new, optimized metaheuristic was used in this study to present an effective CNN based on the previously described cases.

## 6. The Modified Thermal Exchange Optimizer

### 6.1. The Concept of Newton Law of Cooling

Heat transfer that occurs simultaneously with the movement of a fluid is called convection heat transfer. Depending on the process, heat transfer is divided into two categories: free and forced. In free movement, the energy transferred is due to natural factors such as Archimedes' force. But in forced displacement, external forces such as a pump or fan cause the fluid to move. The heat transfer analysis is complex due to the simultaneous process of thermal conductivity and fluid motion. The higher the fluid velocity, the higher the heat transfer rate. The transfer heat transfer velocity can also be expressed using Newton's law of cooling by the following formula:

(13) $$\begin{array}{c} \dot{Q}=\beta \times A\times \left(T_{s}-T_{a}\right), \end{array}$$

where *A* describes the surface of the body that transfers heat, *Q* determines the heat, *α* signifies the coefficient of the heat transfer that relates to numerous cases like surface state, heat transfer mode, and object geometry, and *T*_*b*_ and *T*_*a*_ represent the body and the ambient temperatures.

According to the above equation, heat losing time is *β* × *A* × (*T*_*a*_ − *T*) *dt* that defines reserved heat changing once the temperature *dT* falls, i.e.,

(14) $$\begin{array}{c} V\times \rho \times c\times dT=-\alpha \times A\times \left(T-T_{b}\right)dt, \end{array}$$

where *V* represents the volume (m^3^), *c* defines the specific heat (J/kg/K), and *ρ* describes the density (kg/m^3^). Therefore,

(15) $$\begin{array}{c} \frac{T-T_{b}}{T_{\text{eh}}-T_{b}}=\exp\left(\frac{-\beta \times A\times t}{V\times \rho \times c}\right), \end{array}$$

where *T*_eh_ describes the early high temperature. By considering the (*α* × *A* × *t*)/(*V* × *ρ* × *c*), a time-independent value, i.e.,

(16) $$\begin{array}{c} \zeta =\frac{\alpha \times A}{V\times \rho \times c}. \end{array}$$

That *ζ* is a constant, the main equation can be reformulated as follows:

(17) $$\begin{array}{c} \frac{T-T_{b}}{T_{eh}-T_{b}}=\exp\left(-\zeta t\right). \end{array}$$

Accordingly,

(18) $$\begin{array}{c} T=\left(T_{\text{eh}}-T_{b}\right)\times \exp\left(-\gamma t\right)+T_{b}. \end{array}$$

### 6.2. Thermal Exchange Optimization Algorithm

After explanations about the concept of Newton's law of cooling, it is time to explain the concept of optimization and the relation of the Newton law of cooling and the optimization [13]. Generally, optimization contains all techniques that are used for finding the best solution for optimization problems. Several methods of optimization techniques have been introduced for this aim. Classic methods give exact results for the optimization problems, but recently, by increasing the complexity of these problems, the ability to solve the problems with these algorithms is decreasing. Metaheuristics are intelligent algorithms that are used to find the optimal solution and resolve the before mentioned issues [14, 15]. Metaheuristic algorithms are approximation optimizers that have solutions to exit the local optimization and proper for a wide range of problems. Metaheuristic algorithms are an inspiration of various phenomena from the nature, behaviors of animals, breeding, to human societies and use these conceptions to simulate an approach for solving the optimization problem. Several kinds of metaheuristic algorithms have been proposed in recent years [16, 17], for example, biogeography-based optimization [18], elephant herding optimization [19], ant lion optimizer (ALO) algorithm [20], equilibrium optimizer [21], world cup optimizer [22], and Thermal Exchange Optimizer (TEO) [23].

Here, an enhanced design of the TEO algorithm is presented to provide more ability for this algorithm in terms of accuracy and consistency. The TEO algorithm is an inspiration of the temperature performance of the objects and their position which is exchanged between warm and cold portions to indicate the updated positions. In the TEO optimizer, the individual is split into two parts. One group is the candidates that are considered as cooling substances, and the other group is considered as the environment, and then, the reverse process has been made.  Figure 4 shows the pairs of transfer objects.

The algorithm begins with a predefined number of random individuals as the initial solutions are as follows:

(19) $$\begin{array}{c} T_{j}^{0}=\underline{T}+\theta \times \left(\overset{¯}{T}-\underline{T}\right),\\ j=1,2,\cdots ,n, \end{array}$$

where *θ* denotes a random magnitude in the range [0, 1], *T*_*j*_^0^ signifies the algorithm early population for the *i*^th^ object, and $\underline{T}$ and $\overset{¯}{T}$ stand for the minimum and the maximum limitations.

After achieving the cost value of the generated candidates, *T* number of the best cost individual positions is saved as *Thermal Memory* (TM) to provide higher efficiency with lower complexity to the algorithm. The *TM* individuals are then combined to the individual, and the equal number of worst candidates is then taken out.

To provide more understanding, consider Figure 5. *T*_1_ describes the environment object for *T*_(*n*/2)+1_ cooling object, and contrariwise. If the object is less than *ζ*, the temperature exchanges gradually. *ζ* is formulated as follows:

(20) $$\begin{array}{c} \zeta =\frac{\text{Cos}\left(\text{object}\right)}{\text{Cos}\left(\text{worst object}\right)}. \end{array}$$

Time is another term in the simulation of the optimizer that is related to the number of iteration. This term is obtained by the following equation:

(21) $$\begin{array}{c} t=\frac{\text{iteration}}{\mathrm{Max}.\text{iteration}}. \end{array}$$

To improve the global searching of the algorithm, the environmental temperature changing is considered that is formulated as follows:

(22) $$\begin{array}{c} T_{i}^{e}=\left(1-\left(\alpha_{1}+\alpha_{2}\times \left(1-t\right)\times \delta \right)\right)\times {T_{i}^{\prime }}^{e}, \end{array}$$

where *δ* describes a random number between 0 and 1, *T*_*i*_′^*e*^ represents the preceding temperature of the object modified by *T*_*i*_^*e*^, and *α*_1_ and *α*_2_ represent the control variables, respectively.

Finally, the new position for the object temperature is achieved by the following:

(23) $$\begin{array}{c} T_{i}^{N}=T_{i}^{e}+\left(T_{i}^{\text{old}}-T_{i}^{e}\right)\exp\left(-\zeta t\right). \end{array}$$

The algorithm also defines whether a component changes in the cooling objects or not. This has been stimulated by a term, called Pr. The Pr contains some individuals that are compared with *R*(*i*) which is a random value in the range [0, 1]. If *R*(*i*) is less than Pr, one dimension of the *i*^th^ candidate is randomly chosen and the magnitude is reformulated as given in the following:

(24) $$\begin{array}{c} T_{i,j}={\underline{T}}_{\text{j}}+\delta \left({\overset{¯}{T}}_{\text{j}}-{\underline{T}}_{j}\right)\exp\left(-\zeta t\right), \end{array}$$

where *T*_*i*,*j*_ describes the variable number *j* of the individual number *i* and ${\underline{T}}_{j}$ and ${\overset{¯}{T}}_{\text{j}}$ represent the lower and the higher limitations of the parameter number *j*, respectively. The algorithm is then terminated when the stopping criteria have been reached.

### 6.3. Advanced Thermal Exchange Optimizer

Although the Thermal Exchange Optimizer has a proper speed in solving the problems, it may be trapped in the local optimum point once solving complex and nonlinear optimization problems. Due to this problem, here, an advanced design of the TEO algorithm is designed and suggested to develop the search power of the original TEO algorithm and to resolve the mentioned issue. The movement of the worst individual in the groups (*T*_*w*_) is improved in each iteration of the local search in the Advanced Thermal Exchange Optimization (ATEO) algorithm. First, an exchange vector is generated for the worst solution in each iteration:

(25) $$\begin{array}{c} T_{i}^{a}=T_{b}+\gamma \times \left(T_{r1}-T_{r2}\right), \end{array}$$

where *T*_*b*_ signifies the best solution achieved by the current iteration, *T*_*r*1_ and *T*_*r*2_ represent two dissimilar agents that are randomly chosen from the population in each group, and *γ* describes the exchange coefficient to determine the differences range between *T*_*r*1_ and *T*_*r*2_.

By considering the above condition, the value of the *j*^th^ parameter of the vector *T*_*i*_^New^ in the following iteration is achieved as follows:

(26) $$\begin{array}{c} T_{i}^{\text{New}}=\left\{\begin{array}{cc} T_{i}^{a} & \text{if }\mathrm{rand}<\text{CG},\\ T_{i}^{N} & O.W., \end{array}\right. \end{array}$$

where CG signifies the general intersection constant between 0 and 1 and rand signifies a random constant in the range of [0, 1]. If the cost value of the new solution has proper value in comparison to the preceding solution, the new individual substitutes the former one; else, it will be kept with no changes.

To give a proper result with the TEO algorithm, the population size should be selected wisely. Indeed, population size is a term to define the number of individuals (candidates) that are randomly generated and tested on the objective function to get the best solution. However, this case is one of the difficult parts of all metaheuristics [24]. Here, a self-adaptive mechanism is used for adjusting this case in each iteration. The main characteristic of the self-adaptive mechanism is that it regulates the population size automatically in each iteration with no user intervention [25]. Based on this mechanism, the initial population size before starting the algorithm main loop is considered as follows:

(27) $$\begin{array}{c} \text{PS}=10\times D, \end{array}$$

where PS signifies the population size and *D* describes the problem dimensions. So, the new population size is achieved by the following:

(28) $$\begin{array}{c} {\text{PS}}^{\text{New}}=\text{round}\left(\text{PS}+\text{rnd}\times \text{PS}\right), \end{array}$$

where rnd defines a random magnitude in the range [-0.5, 0.5].

The population size will increase or decrease by up to half the current population size. If the population size obtained for the next iteration increases compared to the population size in the former iteration (PopSize_new_ > PopSize), then all members of the present individual are kept unchanged.

Once the population size in the former iteration decreases compared to the population size (PopSize_new_ < PopSize), the best members of the present population are kept and the weak members have been discarded. If the size of the population does not change (PopSize_new_ = PopSize), so there will be no population changing. Finally, if the new population size reduces from the problem dimensions (PS^New^ < *D*), then the population size becomes equal to the problem dimension.

### 6.4. Algorithm Verification

After designing and introducing the proposed Advanced Thermal Exchange Optimization (ATEO) algorithm, the performance of the method should be analyzed to ensure its ability in use in our purpose.

The present work uses the Single Objective Bound Constrained Numerical Optimization (CEC2020) benchmark standard benchmark in 20 dimensions to analyze the effectiveness of the method; in other words, each faction has 20 decision variables that should be optimally selected. The CEC2020 is known as one of the latterly introduced benchmark functions for analyzing optimization problems. The termination criteria, including the maximum number of the calculation of the fitness function and the minimum error value, are set 1*e*7 and 1*e* − 8, respectively. The constraint of the decision variables is in the range [−100, 100], and 35 independent runs have been established for giving a reliable result. The formulation for each equation can be found in [26]. To provide an appropriate analysis for the suggested algorithm, a comparison of its results with some latest algorithms including blackhole (BH) [27], multiverse optimize (MVO) [28], spotted hyena optimize (SHO) [29], and original Thermal Exchange Optimization (TEO) [23] algorithm has been performed.  Table 2 indicates the parameter setting of the compared algorithms.

During the simulations, for all of the compared algorithms, the population size is equal to 150. To analyze the algorithms' behavior, the mean magnitude and the (mean) and the standard deviation value (Std) have been extracted from the results.  Table 3 discusses the achievements of the algorithms applied to the CEC2020 benchmark sets.

As seen in Table 3, the scores of the analyzed algorithms have been shown. It is clear from the results that in some test functions, the suggested ATEO algorithm escapes the local optimum and found the optimal value. Here, the mean value is employed to consider all of the runs for the algorithm, although the minimum value of the algorithms gives too better or even incomparable results. The minimum value of “Mean” for the proposed ATEO algorithm against the other compared algorithms indicates its higher accuracy to find the minimum value. On the other hand, the minimum value of “Std” for the proposed ATEO algorithm state's better reliability of the proposed algorithm than the comparative methods for the studied CEC2020 benchmark function.

## 7. Classification

With the advances made in the field of imaging and production of high-resolution digital images, the need for accurate image classification is felt so that one of the most basic parts of image processing is image classification. The important point in image classification is providing a method with high accuracy. Taking into account the above-mentioned reasons, backpropagation is in the form of preparing in the CNN mostly. We also clarified why different methods have been proposed to overcome it because of certain major drawbacks of the backpropagation method. Here, the proposed Advanced Thermal Exchange Optimizer (ATEO) is developed and used to reduce the proper and output magnitude by the selection of suitable network weights replacing backpropagation in CNN for mean square error (MSE). The MSE can be mathematically described by the following equation:

(29) $$\begin{array}{c} \text{MSE}=\frac{1}{T}\overset{N}{\underset{j=1}{\sum }}\overset{M}{\underset{i=1}{\sum }}{\left(y_{j}^{i}-d_{j}^{i}\right)}^{2}, \end{array}$$

where *M* and *N* represent the value of the output layers and the data, respectively, and *y*_*j*_^*i*^ and *d*_*j*_^*i*^ define the obtained and the proper magnitudes for *j*^th^ unit in the output layer of the CNN in time *t*, respectively.

## 8. Simulation Results

This study presents an efficient and automated method for brain tumor detection by combining deep neural networks and metaheuristics. The technique involves image preprocessing, image segmentation, extraction of features, and then classification. Based on digital mammogram images, the process is validated.

### 8.1. Dataset Description

To verify the accuracy and the ability of the suggested method, it is performed to a standard mammographic benchmark database, known Image xAnalysis Society Digital Mammogram Database (MIAS) [30]. The MIAS database is compiled by UK researchers to support researchers involved in working on mammogram images. The database includes 322 number of 1024 × 1024 digital mammography images that are taken from the UK National Breast Screening Program. The MIAS database also includes correct labels which are obtained with the help of experts. This database has been gotten available by the Pilot European Image Processing Archive (PEIPA) at the University of Essex. Figure 5 shows some examples of the MIAS database mammography images.

### 8.2. Simulations

By performing the discrete wavelet transform to the image and using decomposition of LL and HL characteristics from it, the GLCM characteristics are achieved by the wavelet decomposition's extracted levels. Then, the features are combined with the optimized CNN-based classifier that is arranged for the final detections. As mentioned before, five features including homogeneity (*H*), correlation (Cr), contrast (CN), energy (*E*), and entropy (ER) are employed to the LL and HL subband levels on the image.  Table 4 illustrates the feature extraction for preparing data.

Also, Table 5 illustrates the feature extraction for the testing data.

For more clarification of the proposed automatic system, it is validated by three measurement indicators, precision, sensitivity, and specificity that are formulated in the following:

(30) $$\begin{array}{c} \text{Accuracy}\left(\%\right)=\frac{\text{TP}+\text{TN}}{\text{TP}+\text{FP}+\text{FN}+\text{TN}},\\ \text{Sensitivity }\left(\%\right)=\frac{\text{TP}}{\text{TP}+\text{FN}},\\ \text{Specificity }\left(\%\right)=\frac{\text{TN}}{\text{FP}+\text{TN}}, \end{array}$$

where TN, TP, FN, and FP represent Truly Negative, Truly Positive, False Negative, and False Positive, respectively.

To proper validation of the suggested technique, it was compared with three latest techniques including Multilayer Perceptron (MLP) [31], Multiple Instance (MI) [32], and Transfer Learning (TL) [33].  Figure 6 shows the comparison results between the suggested pipeline Advanced Thermal Exchange Optimization algorithm-based methodology and the mentioned methods applied to the MIAS database.

Based on Figure 6, the suggested ATEO-based methodology with a 93.79% accuracy rate has the highest precision, and the method of MI, TL, and MLP with 82.91%, 82.91%, and 81.99% is placed in the later ranks. Furthermore, the specificity of the suggested method with 67.7% provides the best achievements than the other compared methods. Finally, the total achievements display optimal results for the suggested technique to automatic breast cancer diagnosis.

## 9. Conclusions

Breast cancer has been a cause of death in women in the last decade; the rate of breast cancer is increasing worldwide. This cancer is common cancer detected in women, and death from breast cancer is more common in women between the ages of 15 and 54. In recent years, much research was performed on mammographic images to be able to diagnose cancerous tumors ignoring the intervention of a person by image processing methods and computer programming. The present study presented a computer-aided diagnosis system for automatic detections of breast cancers. The mammogram images were first preprocessed based on image contrast enhancement and noise reduction to improve and prepare the image for the next steps. Afterward, a method based on color space was used for image segmentation that is followed by mathematical morphology. To achieve the main characteristics of the mammogram images, a combined gray-level cooccurrence matrix (GLCM) and discrete wavelet transform (DWT) was applied to the processed images. Finally, a new optimized version of convolutional neural network (CNN) and a new improved metaheuristic, called Advanced Thermal Exchange Optimization algorithm, was applied for features' categorization. Simulation achievements of the suggested technique were finally compared with three other techniques including Multilayer Perceptron (MLP), Multiple Instances (MI), and Transfer Learning (TL) applied on the MIAS mammogram database to show its superiority.

## Figures and Tables

**Figure 1:** The statistical information of the cancers (a) and cancer deaths (b) in 2019 [2].

**Figure 2:** Several instances of the breast segmentation of images depending on the approach suggested: (a) basic image and (b) segmented image.

**Figure 3:** An overview of convolutional neural network architecture.

**Figure 4:** The pairs of transfer objects.

**Figure 5:** Some examples of the MIAS database mammography images.

**Figure 6:** The comparison results between the suggested pipeline ATEO-based methodology and the mentioned methods applied to the MIAS database.

**Pseudocode 1:** The pseudocode of the Otsu algorithm.

**Table 1:** Five GLCM features extracted from the samples.

Feature name	Mathematical equation
*Contrast*	$\overset{m-1}{\underset{i=0}{\sum }}\overset{n-1}{\underset{j=0}{\sum }}{\left(i-j\right)}^{2}f\left(i,j\right)$
*Entropy*	$-\overset{m-1}{\underset{i=0}{\sum }}\overset{n-1}{\underset{j=0}{\sum }}\log_{2}f\left(i,j\right)$
*Energy*	$\sqrt{\overset{m-1}{\underset{i=0}{\sum }}\overset{n-1}{\underset{j=0}{\sum }}f^{2}\left(i,j\right)}$
*Correlation*	$\frac{\sum_{i=0}^{m-1}\sum_{j=0}^{n-1}\left(i,j\right)f\left(i,j\right)-\mu_{i}\mu_{j}}{\sigma_{i}\sigma_{j}}$
*Homogeneity*	$\overset{m-1}{\underset{i=0}{\sum }}\overset{n-1}{\underset{j=0}{\sum }}\frac{1}{1+{\left(i-j\right)}^{2}}f\left(i,j\right)$

**Table 2:** The variable setting of the compared optimizers.

Algorithm	Parameter	Value
BH [27]	*a*	[0, 1]
	Number of stars	100
MVO [28]	Traveling distance rate	[0.6, 1]
	Wormhole existence prob.	[0.2, 1]
SHO [29]	$\overset{⟶}{M}$	[0.5, 1]
	$\overset{⟶}{h}$	[5, 0]

**Table 3:** The comparison achievements between the suggested ATEO algorithm and the other compared algorithms on the CEC2020.

		ATEO	TEO [23]	BH [27]	MVO [28]	SHO [29]
F1	Mean	7.38*e*8	5.83*e*11	4.22*e*15	8.37*e*13	9.07*e*15
	Std	1.29*e*8	6.19*e*10	5.13*e*13	4.38*e*11	5.46*e*11
F2	Mean	5.79*e*1	9.67*e*2	4.67*e*3	1.76*e*4	4.46*e*6
	Std	4.31*e*1	2.84*e*2	3.82*e*2	6.37*e*2	2.08*e*5
F3	Mean	2.08*e*1	6.92*e*2	9.37*e*2	5.17*e*2	4.83*e*5
	Std	1.46*e*0	3.27*e*0	4.28*e*1	8.09*e*1	6.17*e*4
F4	Mean	0.00	6.15*e* − 10	5.80*e* − 6	4.96*e* − 7	7.67*e* − 6
	Std	0.00	3.48*e* − 11	9.37*e* − 7	4.18*e* − 8	4.08*e* − 8
F5	Mean	1.76*e*2	4.53*e*2	6.37*e*4	6.55*e*3	9.86*e*7
	Std	3.82*e*1	1.27*e*2	5.19*e*3	2.41*e*2	8.19*e*3
F6	Mean	3.29*e* − 1	6.12*e* − 1	8.09*e*0	7.18*e*0	2.96*e*1
	Std	4.13*e* − 1	2.73*e* − 1	3.46*e* − 1	4.82*e* − 2	4.63*e*0
F7	Mean	3.18*e*0	4.16*e*0	8.09*e*1	5.33*e*2	4.29*e*3
	Std	1.24*e*0	1.08*e*0	6.17*e*1	6.81*e*1	2.82*e*2
F8	Mean	7.19*e*1	8.35*e*2	2.19*e*4	5.24*e*5	2.56*e*4
	Std	2.76*e*0	4.37*e*0	3.77*e*1	4.65*e*1	4.07*e*3
F9	Mean	1.96*e*2	3.17*e*2	6.51*e*3	2.85*e*3	5.11*e*4
	Std	1.07*e*1	2.03*e*1	8.09*e*2	6.19*e*1	6.97*e*1
F10	Mean	5.76*e*2	9.83*e*2	9.23*e*3	5.37*e*3	5.17*e*3
	Std	4.27*e* − 1	5.94*e* − 1	2.60*e*0	1.93*e*1	6.93*e*1

**Table 4:** The feature extraction for training data.

#	*H*	CR	*E*	CN	ER
1	0.816	0.173	0.794	0.257	0.298
2	0.757	0.038	0.996	0.047	0.264
3	0.869	0.046	0.957	0.032	0.317
4	0.806	0.042	0.896	0.031	0.376
5	0.794	0.041	0.987	0.135	0.395
6	0.843	0.010	0.917	0.009	0.219
7	0.585	0.057	0.967	0.037	0.293
8	0.810	0.007	0.968	0.011	0.417
9	0.594	0.068	0.979	0.028	0.294
10	0.704	0.041	0.968	0.046	0.407

**Table 5:** The feature extraction for the testing data.

#	*H*	CR	*E*	CN	ER
1	0.794	0.072	0.794	0.047	0.272
2	0.758	0.053	0.856	0.012	0.311
3	0.786	0.032	0.851	0.046	0.347
4	0.865	0.029	0.783	0.019	0.215
5	0.749	0.028	0.764	0.018	0.337
6	0.708	0.029	0.886	0.029	0.318
7	0.819	0.017	0.895	0.053	0.319
8	0.693	0.022	0.851	0.031	0.420
9	0.649	0.034	0.817	0.050	0.433
10	0.684	0.069	0.963	0.079	0.351

## Data Availability

The database for analysis is based on MIAS (the mammographic image analysis society digital mammogram database) which can be obtained as follows: http://peipa.essex.ac.uk/info/mias.html.
